# Development of Educational Communication Path of Journalism in Colleges and Universities in the Era of Mobile Communication

**DOI:** 10.1155/2022/6865273

**Published:** 2022-01-28

**Authors:** Xiaoman Xu, Chunxia Liu

**Affiliations:** ^1^Hebei University, Baoding, 071000 Hebei, China; ^2^Handan University, Handan, 056000 Hebei, China

## Abstract

The development of journalism has a huge impact on mobile communication technology and media ecology. Especially in terms of information dissemination, it not only allows people to better obtain the content they are interested in but also provides media workers with more ways to understand their own needs, meet the needs of audiences, and enhance competitiveness. Therefore, in order to enhance the development space of the journalism major, this article studies the communication development path of this major in colleges and universities in the era of mobile communications. This article mainly uses case analysis method, data method, and investigation method to study the development of journalism education in colleges and universities. The survey results show that 21 people believe that the authenticity of news is an indispensable item in teaching. Therefore, the education and communication development of journalism majors in colleges and universities cannot ignore the principle of authenticity. There are 18 people who think it is necessary to tie their majors with the Internet, indicating that colleges and universities can use the Internet platform to teach journalism.

## 1. Introduction

The rapid development of mobile communication technology has enabled people to obtain information more conveniently in their lives, and at the same time, profound changes have taken place in the communication path of journalism education in colleges and universities. First of all, from the perspective of teaching methods, the traditional classroom teaching mode can no longer meet the society's demand for talent training under the current era. Secondly, from the perspective of course content, “paper-based” textbooks have gradually increased and been continuously updated and improved. In terms of media technology again, the rapid development of mobile communications and becoming one of the mainstream media are driving the rapid and healthy development of my country's information industry and media industry. Therefore, it is necessary to study the new development path of journalism. Mobile communication refers to the communication mode between mobile users and fixed point users or between mobile users, a communication in which one or both parties are in motion, including land, sea, and air mobile communication. The frequency bands used are low frequency, intermediate frequency, high frequency, VHF, and UHF. The mobile communication system consists of mobile station, base station, and mobile switching office.

There are many studies on the communication channels of journalism education in colleges and universities. For example, Zhou Song said that the advent of the era of media convergence has brought tremendous changes and shocks to the entire media industry. Under the new communication environment, my country's college journalism education has more thoughts on the reform and exploration of development paths [1]. Tingting and Qiushi said that in the context of the new era, the picture of “news communication” is becoming clearer and clearer. Since the emergence of news dissemination in colleges and universities, it follows the development of the times and the development of college students to continuously adjust the practical goals and dissemination paths [2]. Dongxue and Danyang believe that college media is the carrier of college information dissemination. The continuous popularization of mobile communication equipment has made new media appear on the stage of colleges and universities [3]. Therefore, the key to the development of journalism in colleges and universities lies in the use of communication networks to carry out various types of specialization. The subject of this article is a research hotspot, which is worth exploring. There are differences between media and media: media is the carrier, medium, or channel needed for information dissemination. Media is a combination of media+content system, with system support such as back-end content architecture, production process, and editing and reading interaction. Therefore, in addition to mastering the processing technology of multiple media, we must have a content system to support the processing process and finally realize the good combination of content and channel.

This article first elaborates on mobile communications and then studies the changes, challenges, and advantages of news broadcasting in the Internet era. Then, this article studies the status quo and problems of journalism education under media convergence. After that, I analyzed the development direction of journalism and took MOOC as an example to explore the new direction of journalism teaching. Finally, a questionnaire survey was conducted and the results were obtained. Media integration is not only the diversification of information collection channels and communication channels. What is important is that media staff can comprehensively sort, refine, and process according to the original materials of multimedia, quickly convey information through the characteristics of different media communication, express the truth behind the event, and restore the whole picture of the news, so as to improve the quality and depth of news reports.

## 2. The Development of the Communication Path of Journalism Education in Colleges and Universities in the Era of Mobile Communication

### 2.1. The Era of Mobile Communication

Since its birth, mobile communication networks have continuously integrated various cutting-edge technologies in communication research, aimed at building an intelligent society with “Internet of Everything”. From 1G to 4G is mainly to ensure the mutual communication between people, as well as the data transmission of a small number of Internet of Things devices. With the rapid development of the information age, on the one hand, the large-scale growth of Internet of Things devices and changes in service content. The original Internet of Things is mainly a small fixed sensor device such as smart meter reading that unilaterally uploads a small amount of data to the base station periodically. The use scene is single, and the interactive content is simple. In 5G, the application requirements of the Internet of Things are closer to all aspects of people's lives, more intelligent, and more pursuit of good interaction between people and peripheral smart devices, that is, let the Internet of things devices have a “human brain” and respond in a complex external environment for different needs of people. The basic characteristics of the Internet of things from the perspective of communication objects and processes, the information interaction between things, and people and things are the core of the Internet of things. The basic characteristics of the Internet of things can be summarized as overall perception, reliable transmission and intelligent processing. For overall perception, various information of objects can be perceived and obtained by using sensing devices such as RFID, QR code, and intelligent sensor.

#### 2.1.1. 5G Random Access

5G random access needs to meet mass access, reduce access delay and signaling overhead as much as possible, improve the flexibility and autonomy of the UE, and enhance the function of random access. The journalism profession emphasizes timeliness and authenticity. Therefore, in the 5G environment, the speed of information dissemination can reach a faster speed, and the random access of news also needs to keep up with the development of the times [4]. 5g network is a new network mode at present, and its penetration rate is still relatively low, which still needs further research and development. The so-called 5g network refers to the fifth-generation network in the development of mobile communication network. Compared with the previous four generation mobile networks, 5g network shows more strengthened functions in the process of practical application, and theoretically, its transmission speed can reach tens of GB per second, which is hundreds of times that of the 4G mobile network. For 5g network, it shows more obvious advantages and more powerful functions in the process of practical application.

The Markov chain model is widely used in the access control of communication networks and can well simulate the random process of data transmission and backoff.

The Markov chain of discrete time and discrete state is denoted and its state space is denoted. According to the conditional transition probability formula, for any two integers *m* and *w*,

(1) $$\begin{array}{c} O\left\{A_{k+m}=x_{v}\left|A_{s_{1}}=x_{i_{1}},A_{s_{2}}=x_{i_{2}},\cdots A_{s_{h}}=x_{i_{h}},A_{k}=x_{i}\right.\right\}. \end{array}$$

When the transition probability is only related to the time distance *m* and *i*, *vj*, there are

(2) $$\begin{array}{c} O_{iv}\left(k,k+m\right)\Delta O_{i,v}\left(m\right). \end{array}$$

It is said that the transition probability is stationary or homogeneous.

The Markov chain can be defined by transfer matrix and transfer graph. In addition to Markov, the Markov chain may have irreducibility, recurrence, periodicity, and ergodicity. An irreducible and normal recurrent Markov chain is a strictly stationary Markov chain with a unique stationary distribution. The limit distribution of ergodic Markov chain converges to its stationary distribution.

### 2.2. Advantages of News Broadcasting Development in the Era of Mobile Internet

#### 2.2.1. Change

1. The audience is huge. The development of the new era of news media is embodied in the word “movement”, which is not only dynamic in the way of dissemination but also the way of propaganda is dynamic. Whether it is communication space, audience groups, or information services, it is fluid [5]
2. The audience is getting younger and younger

The post-90s and post-00s have witnessed the rise and development of the Internet. With the continuous changes in technology and innovations, the receiving tools of news audiences have become more diversified and modern. These changes include the popularization of smart phones and the popularization of mobile networks. The audience structure presents the development trend of younger, higher income, and higher knowledge [6].

(3) Typed news is more popular, and the frequency is more professional

News can be divided into different sections. Each type of news will be classified and specifically designed, for example, sports news, entertainment news, and social news. Both the diversification of types and the specialization of news are inseparable from mobile communications.

(4) Multimedia terminal, fragmented viewing time

In the era of mobile internet, mobile phones are the mobile devices that accompany us for the longest time every day, and the time we use mobile phones is becoming more and more fragmented. You can read all kinds of news every day with a random tap on your mobile phone, or you can learn about what is happening in society through the broadcast, newspapers, etc.

The multimedia system terminal consists of two parts: multimedia hardware system and multimedia software system. The hardware system mainly includes the main configuration of the computer, various external devices, and the control interface card with various external devices (including multimedia real-time compression and decompression circuit). The software system includes multimedia driver software, multimedia operating system, multimedia data processing software, multimedia creation tool software, and multimedia application software.

#### 2.2.2. Challenge

1. Increased types of news and a large amount of information

Because different types of news all want to expand their own sections, the competition is fierce. Moreover, due to the current sharing and contagious nature of information, all kinds of information are expanding. Therefore, if students majoring in journalism cannot handle all kinds of mass information well for publicity, they are likely to be covered by information [7, 8].

(2) The regulatory mechanism is not in place

News published online are sometimes just rumors or appearances. Without checking, the news lacks authenticity. However, the state's supervision of news uploads is not in place, leading to the random spread of fake news following smart devices. Therefore, if journalism students cannot guarantee that what they are revealing is the truth or a gimmick, there is no need to be a journalist [9, 10].

#### 2.2.3. Development Advantages

1. Specialization

After entering the era of mobile internet, the tools of mass media have become increasingly diversified, and the needs of audiences have become increasingly segmented. Information should be divided into multiple levels according to the diverse requirements of the audience, including program settings and content positioning.

(2) Outstanding service features

These need to be more specific and practical to serve the broad masses of people. This feature is also an important means to ensure that the mobile crowd is a loyal audience. We must have the ability to deliver the most accurate and effective information to everyone at any moment, so that the development of journalism can flourish [11–13].

(3) Focus on multiparty cooperation

Different levels of the news section can support each other, not only do the content of their own section but also help the development of other sections of the news.

(4) Regional coverage

The Internet allows news to spread all over the country. Although news has its own characteristics in each region, in addition to receiving local news, people can also learn about news all over the country and even the world.

### 2.3. Status Quo of Journalism Education and Facing Dilemmas

#### 2.3.1. Current Status of Journalism Education

Journalism education in my country's colleges and universities has achieved an extraordinary and leap-forward development. However, the blind expansion behind the prosperity and development inevitably hides the crisis. Journalism colleges have problems such as lack of professional teachers, irrational structure of teaching staff, incomplete talent training system, outdated models and methods, equipment and other teaching resources, and serious lack of training and practice bases. This leads to a decline in the quality of talent training and lower talent competitiveness and sustainable development capabilities.

The number of various types of media has stabilized, the talent team has become younger, and the demand has become saturated. As the country implements the exit mechanism of newspapers and periodicals, some newspapers and periodicals will withdraw from the market. As cultural undertakings undergo reforms, various media will further integrate and optimize resources. Media is further integrated. In order to improve efficiency and effectiveness, the professional skills and quality requirements of editors and editors will be higher, the entry system will be more stringent, and some media may also face layoffs.

#### 2.3.2. Difficulties Faced

1. The training goals are vague and convergent, and the teaching concepts are backward

The training goals and curriculum settings of journalism convey a message—because of traditional newspaper education, the completion of teaching tasks is the old concept of cultivating talents. At present, great changes have taken place in the form of media and the ecological environment. New media are emerging one after another, and the integration of media is deepening. But there are still many teachers who do not recognize this change, or even understand journalistic skills.

(2) Less capital investment, lack of internal and external resources

Journalism and communication majors are regarded as engineering subjects in liberal arts, which shows the importance of skills to journalism students. At present, many local colleges and universities have leaders who believe that journalism education means training students' ability to collect, write, edit, and comment. In recent years, local colleges and universities have increased their infrastructure construction and the funds have been tight, so they are even more reluctant to invest in the construction of liberal arts laboratories. The construction of laboratories and practice bases is an important factor restricting the development of journalism in colleges and universities.

(3) The teachers are relatively weak, and the media background experience is less

The lack of professional teachers is another bottleneck in the development of journalism in local universities. Some colleges and universities do not even have a teacher with background knowledge of journalism. Most teachers only come into contact with professional knowledge of journalism when they get the textbooks for the first time, let alone the accumulation of academic qualifications and skills. Many colleges and universities have also tried to invite experienced media workers to teach in the school by way of part-time professors or external appointments. However, due to the unresolved identity problem, the busy work of the media workers, the need to improve teaching skills, and the unresolved teaching time and quality, the expected results have not been achieved.

(4) The curriculum system is unreasonable, and the students are not expert or master

The setting of the curriculum system is one of the important manifestations of the teaching system and teaching guiding ideology. Because of the lack of professional teachers, in actual teaching, there are more literature courses and fewer courses to adapt to media integration. The current media needs compound talents, which need a generous knowledge structure to support. The decrease in employment of a large number of journalism graduates in the industry will directly affect the reputation of journalism and communications majors.

The weaknesses of journalism and communication include lack of exclusive research content, lack of personalized service function, and simple expression form. From the perspective of Internet development, database and search engine will be the main trend. For example, overseas media websites not only provide the latest articles but also provide search and query of previous articles. At present, domestic media channels lack database support and are difficult to query and search.

### 2.4. The Integration of New and Old Media Promotes the Development of News Dissemination

1. “Integrated News” came into being

With the emergence of the convergence of old and new media, “converged news” came into being. The prepared text reports can be used in traditional media newspapers and can also be provided to new media networks and mobile phones. The joint action of the new and old media in the collection and release of news information has not only realized resource reorganization and resource sharing and reduced the investment of manpower, capital, and equipment but also promoted the optimization and adjustment of the organizational structure and work flow of different media.

(2) Public participation in news dissemination

With the integration of new and old media, news reporters are no longer just professional reporters. Whether they are volunteers or tourist audiences, they may become the main body of news sources and news dissemination. The content of new online media and traditional media complement each other, which is also manifested in the sharing of news events and the cooperation of thematic columns.

(3) Promote news dissemination and entertainment

The so-called entertainment of news dissemination, in addition to the pursuit of beauty and artistry in terms of expression methods, mainly means that news dissemination does not focus on social events itself but pays special attention to entertainment news related to people, events, and things.

(4) Changing the way journalists work

Under the continuous development trend of the integration of new and old media, the boundaries between various media are becoming increasingly blurred, and the methods and channels of communication are unprecedentedly rich. Therefore, higher requirements are placed on the quality of journalists themselves. Journalists must follow the trend and strive to change working methods, comprehensive use of various techniques and techniques, to provide audiences with a full range of multimedia and three-dimensional news services.

### 2.5. Journalism Education Reform

#### 2.5.1. The Value of MOOC to the Reform of Journalism Education

1. Realize teaching students in accordance with their aptitude and provide learners with personalized choices

In the information society, learners of journalism and communication can choose different types of news on MOOC according to their personal interests after mastering the necessary knowledge through the core courses taught in traditional universities with conceptual maps of the subject. The marginal courses of communication disciplines, or courses of other disciplines, are compensations for the imbalance of knowledge and ability, theory and practice, instrumental rationality, and humanism that have emerged in industrialized higher education. From a microperspective, MOOC can aim at the shortcomings of overdivision and overdivision of majors and promote the integration of subjects such as arts, sciences, and arts in the individual knowledge pedigree, so that learners have stronger employment competitiveness.

(2) Integrate global resources and enrich the education resources of journalism and communication

In the integration of human resources, MOOC can fully break the admission system of college teachers. It can be said that as long as someone is willing to listen, anyone can become a teacher on the Internet. Second, for the integration of subject resources, the information society requires media practitioners not only to have the ability to collect and report news facts but also to have high information integration and analysis capabilities. Journalists need to accurately judge the news value of a certain social phenomenon or event and conduct in-depth analysis and comment on this particular phenomenon, event, or topic. MOOC provides a large platform that integrates resources of various disciplines.

(3) Open the teaching system and expand the training methods of journalism and communication talents

First, for the openness of content, being open does not only mean that MOOC has no standardized and immutable teaching content. Learners can share learning resources, discuss, and communicate with others. Second, for the openness of the method, MOOC provides a reference for setting up learning expectations. Learners set their own learning goals, learning time, and learning location, and freely decide how much energy to invest. Third, for the openness of teaching evaluation, with the help of computer technology, MOOC can monitor the entire learning process of learners. The computer can accurately evaluate learners' learning frequency, learning duration, and learning speed and provide feedback to learners.

From the structural and functional level, MOOC helps to build a basic framework for learning content, establish different learning goals for a personalized personal knowledge pedigree, and provide it with multiple and operable ways to achieve goals.

## 3. Questionnaire Survey

### 3.1. Questionnaire Design

The topic of this questionnaire is the development of journalism education in colleges and universities. The content of the questionnaire was designed by the five members of the group to think together. Questions in the questionnaire include the following general aspects:

1. Intention to study and study in journalism major
2. Journalism students' views on journalism employment
3. The opinions of journalism majors on the teaching methods they have learned
4. What methods can be used to learn journalism
5. What are the principles that journalism focuses on?

### 3.2. Questionnaire Process

The questionnaire process lasted a week in total, and the subjects of the survey were junior journalism students who were about to enter their senior year. A total of 50 questionnaires were distributed in this round of survey, with a total of 50 invitees. The way to fill in the questionnaire is to fill out the questionnaire offline. 50 questionnaires were returned, and 48 questionnaires were effectively filled out, with an effective response rate of 96%. After collecting the questionnaire, the questionnaire was organized. The types of questionnaire design include structured and unstructured. The structured questionnaire, also known as the closed questionnaire, limits the answers to the questions in advance and allows selection only within the scope limited by the questionnaire. The unstructured questionnaire, also known as open questionnaire, is composed of free questions, which are nonfixed answers.

### 3.3. Questionnaire Statistics

After sorting out the questionnaires, the two of them will input the data into the computer and analyze the data.

## 4. Analysis of Survey Results

### 4.1. Intention to Study and Study in Journalism

In response to the intention of journalism students for postgraduate entrance examinations, the result is that more boys than girls want to continue their in-depth study, see Table 1 for details.

As shown in Figure 1, according to the choices of boys and girls, we can find that 38% of people want to continue their in-depth study of journalism. However, 31% have only thought about it without actual action, indicating that the in-depth study of journalism is confused for students.

### 4.2. Analysis of the Sense of Identity of Journalism Students

According to the survey results, this article has done an overall data analysis from the recognition of professional cognition, emotion, environment, and employment direction. The average ranking of journalism students' recognition of these four aspects is the professional environment first, professional emotions last, professional employment tendency second, and professional cognition third, as shown in Table 2.

As shown in Figure 2, we can see that in the standard deviation, the overall level is not high. Students' recognition of majors depends on the employment situation of journalism majors. The lower professional emotional score is because many students studying journalism nowadays are not for the purpose of passion.

### 4.3. Teaching Direction and Principles of Journalism

With the development of mobile communications, the teaching and dissemination methods of journalism can be carried out from the Internet, practical exercises, basic knowledge training, and resource sharing. The details are shown in Table 3.

As shown in Figure 3, we can judge that authenticity and objectivity are the most important issues for journalism professionals. Secondly, the timeliness of news is also very important. In resource sharing learning, the authenticity of news needs to be guaranteed. When teaching on the Internet, you need to be objective at all times and conduct a rational analysis of things in the news.

Colleges and universities should build a scientific, reasonable, and relatively stable quality management and evaluation system around the school running ideas, talent training objectives, and the needs of employers of journalism and communication majors. Through the omnidirectional, hierarchical, and normalized quality monitoring and management of teaching operation, teaching process, teaching effect, teaching funds, facility construction, teaching reform and research, teaching plan revision, practical teaching reform, students' daily management, graduates' quality tracking, social and employers' evaluation, and other links, we can realize student-oriented. It is a result-oriented quality management goal based on the needs and standards of the employer.

### 4.4. The Choice of Journalism Teaching Methods

From the questionnaire, we can find that students with different levels of academic performance in journalism have different attitudes towards teaching methods. The main teaching methods can be carried out through classroom teaching, electronic equipment, microclass online courses, and books. The specific situation can be seen in Table 4.

As shown in Figure 4, we can see that people with excellent grades do not support classroom teaching and book-based teaching methods, but they have the highest support for microclass learning methods. For those who fail in grades, they are more keen on learning with electronic devices. People with average grades have similar support for different teaching methods.

## 5. Conclusion

In this rapidly developing era of mobile communications, how journalism professionals can use existing communication tools and technologies to learn and understand journalism-related knowledge and carry out practical training is a problem that we need to consider at present. And this article studies the problems of mobile communication and cash journalism, proposes the use of Internet technology in journalism teaching, and cites MOOC tutorials to study the development of journalism. Finally, this paper mainly uses the methods of case analysis, data analysis, and investigation to study the development of Journalism Education in colleges and universities. The survey results tell that journalism education must pay attention to the truthfulness, timeliness, and objectivity of news and use modern network technology to develop journalism. The research results obtained in this paper can provide some reference ideas for the follow-up-related content.

## Figures and Tables

**Figure 1:** Intention to further study in journalism.

**Figure 2:** The overall status of journalism professional identity.

**Figure 3:** Teaching direction and principles of journalism.

**Figure 4:** The choice of journalism teaching methods.

**Table 1:** Intention to further study in journalism.

	Male	Female
Willing	10	9
Unwilling	2	1
It will be all right	6	8
Thought about	8	6

**Table 2:** The overall status of journalism professional identity.

	Professional recognition	Professional emotion	Professional environment	Professional employment tendency	Total score
Mean	3.54	3.31	3.68	3.56	3.52
Standard deviation	0.31	0.63	0.72	0.35	0.31

**Table 3:** Teaching direction and principles of journalism.

	Timeliness	Authenticity	Objectivity
+Internet	5	6	7
+Practical practice	3	5	4
+Basic knowledge	2	4	1
+Resource sharing	4	6	3

**Table 4:** The choice of journalism teaching methods.

	Excellent	Good	Commonly	Flunk
Classroom teaching	1	2	4	3
ED	5	3	2	5
Microclass	6	5	3	2
Books	2	2	4	1

## Data Availability

The data underlying the results presented in the study are available within the manuscript.
